This article has been retracted.

# Dense Convolutional Neural Network for Detection of Cancer from CT Images

**DOI:** 10.1155/2022/1293548

**Published:** 2022-06-20

**Authors:** S. V. N. Sreenivasu, S. Gomathi, M. Jogendra Kumar, Lavanya Prathap, Abhishek Madduri, Khalid M. A. Almutairi, Wadi B. Alonazi, D. Kali, S. Arockia Jayadhas

**Affiliations:** ^1^Department of Computer Science and Engineering, Narasaraopeta Engineering College, Narasaraopeta, Andhra Pradesh 522601, India; ^2^Department of Information Technology, Sri Sairam Engineering College, Chennai, Tamil Nadu 602109, India; ^3^Department of Computer Science and Engineering, Koneru Lakshmaiah Education Foundation, Vaddeswaram, Andhra Pradesh 522502, India; ^4^Department of Anatomy, Saveetha Dental College and Hospital, Saveetha Institute of Medical and Technical Sciences, Chennai, Tamil Nadu 600077, India; ^5^Department of Engineering Management, Duke University, North Carolina 27708, USA; ^6^Department of Community Health Sciences, College of Applied Medical Sciences, King Saud University, P. O. Box: 10219, Riyadh-11433, Saudi Arabia; ^7^Health Administration Department, College of Business Administration, King Saud University, PO Box: 71115, Riyadh-11587, Saudi Arabia; ^8^Department of Mechanical Engineering, Ryerson University, Canada; ^9^Department of EECE, St.Joseph university, Dar Es Salaam, Tanzania

## Abstract

In this paper, we develop a detection module with strong training testing to develop a dense convolutional neural network model. The model is designed in such a way that it is trained with necessary features for optimal modelling of the cancer detection. The method involves preprocessing of computerized tomography (CT) images for optimal classification at the testing stages. A 10-fold cross-validation is conducted to test the reliability of the model for cancer detection. The experimental validation is conducted in python to validate the effectiveness of the model. The result shows that the model offers robust detection of cancer instances that novel approaches on large image datasets. The simulation result shows that the proposed method provides analyzes with 94% accuracy than other methods. Also, it helps to reduce the detection errors while classifying the cancer instances than other methods the several existing methods.

## 1. Introduction

When it comes to breast cancer screening, digital mammography (DM) is the gold standard for women who have no signs or symptoms of the disease. In a diagnostic setting, it has been demonstrated that DM can reduce breast cancer mortality. Rather than seeing clinical images as only graphical representations, advances in medical image analysis have made to consider multidimensional data [1]. It is the process of analyzing medical images to extract information that is of interest to researchers that is referred to as radiomics. With the help of high-throughput computing approaches, it is possible to develop mathematical models and classifiers for diagnostic decision assistance [1], which analyze images and extract a large number of quantitative features. The use of automated image analysis has increased significantly in recent years, owing to intrinsic detected features properties in images.

There are several processes in the quantitative radiomics pipeline that include identifying the region of interest to be explored, and the extraction of quantitative information [2–6]. These characteristics must first be statistically analyzed in order to be used in the development of classification models that reliably anticipate the outcome of the research. It may be necessary to get a variety of mammographic images or to use multiple imaging modalities in order to diagnose an abnormality discovered at DM. A biopsy should be performed if there is a suspicion that a lesion is malignant. According to the results of the study, there are subtle differences between lesions and background fibroglandular tissue, a variety of lesion types, breasts that are not firm, and a relatively modest number of malignancies in the screening sample of women at average risk. As a result of this, there is a considerable amount of diversity both among and between observers [7–10].

To deal with the problem of tissue superposition in mammography, one of the most cutting edge systems for breast imaging has been developed and is being used today. Breast CT, which has been specifically engineered to match the spatial resolution and contrast requirements of imaging [11], can be used to obtain real-time 3D images of the breast in real time. It is possible that radiomic descriptors of aggressiveness and malignancy will be more accurate if tumor characteristics such as morphology and heterogeneity are not layered on top of each other, as is the case with mammography.

Tumors show variable morphological imaging based on their morphology, the definition of their borders, and the variability of voxel intensity [11]. It is necessary to calculate a large number of radiomic features in order to quantify these properties, which results in a large amount of data being recovered from each image. Numerous radiomic properties have a considerable computing cost associated with them, particularly 3D descriptors derived using tomographic imaging [12]. This problem can be somewhat resolved if you think of a tomographic image and perform any analysis. Many studies have shown that using a 2D radiomics technique can get comparable results to radiomic analysis [12] of a straightforward mathematical formulation for radiomic properties [13, 14]. Due to the fact that the information is being supplemented in a 2D manner, it is possible to create robust diagnostic classifiers. Manual classification is inefficient in clinical practice since it requires a significant amount of time. Especially if hundreds of 2D images of each patient must be labelled, this is a major undertaking.

This necessitates the development of automated tumor classification algorithms, which are particularly useful in circumstances when the volume to be segmented is large and of complex shape. The classification task can be trained using supervised deep learning algorithms, which have been shown to produce excellent performance with minimal computing time in previous work on digital mammography, ultrasonography, and magnetic resonance imaging, among other applications. As far as we are aware, there are no supervised classification methods for breast CT, and the DICE similarity performance of these approaches is on average 0.8, with certain scenarios resulting in a DICE of less than 0.7. Further study into the application of deep learning is required in order to segment lesions in breast CT imaging. There has only been a single article on radiomic robustness in dynamically contrast-enhanced breast MRI [12] that has not included any examination of the stability of the descriptors.

A detection module is used in conjunction with lengthy training and testing to construct a dense convolutional neural network model. In order to ensure that the model operates as effectively as possible when utilized in cancer detection, various aspects have been incorporated into the design. Preprocessing of CT scans is required in order to ensure the most accurate classification possible throughout testing and evaluation. The main contribution in this paper, we develop a Dense CNN that aims to classify the tumor cancer datasets from the input data using proposed algorithm. The proposed model is made to undergo series of steps involving preprocessing, feature selection, and predication.

## 2. Related Works

To enhance the accuracy with which tumors or malignancies may be discovered on mammograms, deep learning has recently been used for the categorization of mammograms. Deep learning architectures have been employed in a number of studies to detect and classify breast cancer, and they have shown promising results [11]. They [11] developed a technique of boosted decision tree (DBT) and convolutional neural network (CNN) were tested in the categorization of cancer. The CNN model with the exception that it takes input dimensions into consideration (ROI). The sensitivity of the CNN model was compared to that of the enhanced decision tree model. They contained images that were deemed concerning by radiologists and classified as malignancy since they had a limited number of biopsy-proven cancers, in order to compare outcomes.

The authors [12] proposed a strategy that used two stages of transfer learning to distinguish between DBT images that were normal and those that were abnormal. First, the researchers employed an AlexNet model that had been trained on ImageNet before being fine-tuned with FFDM images. Later, the model is trained on images using the initial weights learned from FFDM images and then tested on images. CNNs are utilized in a second stage to extract features rather than classify them.

They [13] developed VGG19 for feature extraction for the purpose of categorizing them as cancerous or benign, respectively. After each maximum pooling layer, features from the VGG19 model were selected and used. An average pooling technique was employed to reduce the size of the feature dimension. When we wanted to delete traits that were already present, we employed the stepwise feature selection method with the leave-one-out strategy. After that, an SVM classifier with a leave-one-out feature was employed to assess the likelihood of malignancy. The findings of this investigation included the examination of 30 malignant and 48 benign lesions. To build the ROI patches, a mix of FFDM, 2D mammography reconstruction, and slice images were employed in conjunction with DBT z-Stack slice images.

The authors [14] used a deep learning model that has been trained on FFDM images and then modify it to operate with DBT images. These images were divided into four categories according to their FFDM and DBT content. There are four classifications: normal, benign, high-risk, and malignant. Normal is the most common categorization. Normal is the least risky of the four options. The ResNet, with 29 layers, is capable of handling patches of varying sizes as input. FFDM was used to train the model at first, and subsequently, 2D maximum intensity was used. As described by the authors, projections of DBT images were used to train the model.

This work [15] developed a model for identifying masses based on the latent bilateral properties of asymmetric breast tissue to be used for mass classification. The essential element of their thinking is the classification of masses. In the beginning, DBT primary and lateral views were registered using a volume registration system (left and right breast). This was followed by the application of the VOI transform. According to an article [16], feature selection should be performed using a random forest model. They processed images in the data preprocessing module, denoising and augmenting them. The deep CNN produces features that have been learned from z-Stack images. After that, using a MI-RF, the images are categorized as benign or malignant in nature.

According to [17], CNN models were developed. Transfer learning were used in conjunction to get this result. The AlexNet was utilized to train the 2D-T2-Alex model, which was then employed in conjunction with a shallow CNN to distinguish between normal and malignant tissue. In the shallow CNN, one convolutional layer is followed by two 1024 completely linked layers, all of which are implemented with a kernel size and filter depth of 256. When it came to developing new techniques to include the entire DBT volume into models, the same team that had previously worked on the problem came up with new ideas. It was decided to look for techniques to fuse reconstructions of images [18]. They suggested a fusion model with two unique stages of fusion: an early stage and a late stage, which they divided into two categories. According to the findings of this study, the author 3D-AlexNet model outperformed the performance of the early and late fusion stages proposed in their previous research.

This work [19] divided an image into four distinct parts. It all starts with a preliminary classification of the data. In this step, DBT images are utilized to create 2D dynamic visuals that are animated. Every single one of the numerous z-Stack images is blended into a single dynamic image for presentation. The feature extraction process is carried out in two stages, using both 2D dynamic reconstructions and FFDM images. The classifiers used in the fourth stage are based on the features that were extracted in the previous step. The first classifier classifies images based on the characteristics of their dynamic content. It is identified using the second classifier based on the features are concatenated from images. In order to categorize features, the third classifier makes use of FFDM images. The scores of all classifiers were added together using an ensemble approach, which allocates a weight to each classifier in turn. With the use of a CNN model, it was possible to classify the presence of calcification in images reconstructed using a variety of DBT reconstruction approaches. In the shallow network are used in conjunction with each other. While the enhanced multiple parameter iterative reconstruction strategy has an AUC of 0.888, the filtered back projection method has an AUC of 0.857, and the CNN model trained has an AUC of 0.888; the filtered back projection method has an AUC of 0.857.

## 3. Proposed Method

DenseNet [20] is implemented in order to improve image quality while also addressing other performance difficulties. Additionally, the authors provide a new algorithm or pseudocode that may be used to evaluate efficiency and performance in addition to existing mathematical methods. In this paper, a proposed algorithm is made to undergo series of steps involving preprocessing, feature selection, and predication.  Figure 1 depicts the proposed method.

### 3.1. Preprocessing

Preprocessing is the initial step in the image processing process. One such example is the *D* breast cytology image repository, which stores images of breast cytology.

(1) $$\begin{array}{c} ∆D∊\left\{D_{1},D_{2},\cdots D_{n}\right\}, \end{array}$$

where *n* is the images and *D* is the vector function.

Before any further processing can take place, noise is eliminated from the raw cytology images using a powerful Gaussian filtering algorithm. Channels can be used to improve the attractiveness and complexity of an image, as well as to change the surfaces, tones, and other embellishments that are displayed on the image. The following is a characteristic of a Gaussian channel:

(2) $$\begin{array}{c} G_{D}\left(x,y\right)=\frac{1}{2\pi \delta_{D}^{2}}\exp\frac{-\left(x^{2}+y^{2}\right)}{2\pi \delta_{D}^{2}}, \end{array}$$

where (*x*, *y*) is the current image pixel.

### 3.2. Feature Extraction

An estimation is used to characterize the image texture from underlying image, and it is represented by the *E*. It is feasible to distinguish between healthy and malignant cells based on the shape of their nuclei. The number of subsquares utilized to quantify each image textual features.

### 3.3. DenseNet

The result of applying a convolutional network to a single image. It is applied at each layer of the network, which consists of several layers, to perform batch normalization and other nonlinear operations.

### 3.4. ResNet

Traditionally, layer transitions are induced by convolutional feedforward networks, which connect the outputs of preceding layers as inputs to the next layer. When a skip connection is used in conjunction with an identity function, nonlinear transformations are avoided. ResNets have the feature of allowing gradients to flow straight from later layers to earlier layers, which is a significant advantage. Despite this, the summing of the identity function and the output may cause information flow in the network to be slowed.

### 3.5. Dense Connectivity

In order to better optimize information flow between layers, we propose that direct connections be established from any layer to any subsequent layer as another connectivity architecture. As a result, the layer receives feature maps from all of the layers that came before it. The term DenseNet alludes to the high density of connections in this network. For the sake of simplicity, all of the inputs are concatenated into a single tensor for execution.

### 3.6. Composite Function

The research defines a composite function that is made up of three subsequent operations: batch normalization, a rectified linear unit, and a convolution, among others.

### 3.7. Pooling Layers

When the size of feature maps varies, the concatenation procedure becomes impossible. This essential down sampling layer allows convolutional networks to change the size of feature maps as a result of the effects of the down-sampling layer. For the purpose of making downsampling easier, our network has been partitioned into multiple densely connected blocks. Transformations such as convolution and pooling are carried out at transition layers, which can be found between blocks. The layers we used in our experiments included a batch normalization layer, an 11-layer convolutional layer, and a 22-layer average pooling layer.

### 3.8. Growth Rate

In other words, if each function generates feature maps, then the layer will have an equal number of feature maps as the input feature maps. Existing network topologies can have several levels; DenseNet, on the other hand, can have many layers that are extremely small. The hyperparameter *k* indicates the rate at which the network is growing. Because each layer has access to the previous feature maps in its block and, as a result, to the aggregate knowledge of all the other levels in the network, it is possible that this is the case. They can be considered a snapshot of the network general health, similar to that of an image. *K* feature maps from each layer are present in this condition. The rate at which particular layers expand contributes to the inflow of new information into the global state. Traditional networks require state to be duplicated across layers, but global state can be accessed from any tier of the network, unlike global state.

### 3.9. Loss Function

The generalizability and performance of the model are both directly influenced by the loss function that is used. Loss functions in classification and regression are the two most common types of loss functions, and each of these types can be further subdivided if more detail is required. In classification tasks, predicting the class of a sample is a key aspect of the process. As a result, categorization loss is a quantitative measure of the disparity between expected and actual classifications. Rationality is the goal of regression analysis, which is to predict continuously valued outputs from samples of data. The degree of error is determined by comparing the predicted numerical values to the real-world values, which is accomplished through the use of regression loss functions.

An image analysis program for cancer diagnosis using deep learning DBT has three sorts of loss functions: classification, recognition, and classification. Each form of loss function has a different meaning.

## 4. Results and Discussions

The patients in this study ranged in age from 50 to 86 years old, and a total of 69 images were taken, with a total of 93 mass-like lesions being identified in the images. The lesions ranged in size from 4.8 millimeters to 27.0 millimeters in diameter, depending on the main diameter. One hundred and ninety-nine benign tumors were discovered, but only 25 malignant tumors were discovered, and in nine cases, the kind of tumor could not be determined. Through the use of ultrasonography, a total of 49 cysts were discovered, and biopsies verified the presence of 35 solid masses. For each lesion, separate training, validation, and test sets were produced. To avoid bias in the data, we decided in advance the number of cases per kind of lesion that would be included in each dataset before randomly assigning cases to the various datasets.

### 4.1. Data Augmentation

Specifically for this experiment, a single patch of image was obtained in the coronal plane that crossed the mass center in order to perform 2D breast mass classification. This image patch was used to do 2D breast mass classification. The patches we employed had a fixed voxel size of 128 × 128 to ensure that they covered the maximum possible percentage of our dataset. Because deep learning performance is closely connected with dataset size, 58 masses from validation and training sets were each subjected to one of three augmentation techniques. In addition to the coronal patches collected in the previous step, an additional 8 patches are collected in the first augmentation step.

It was decided to take six more diagonals from the imaginary cube by cutting two opposed sides of the imaginary cube into its diagonals using planes of symmetry. Following the implementation of this approach, a total of 522 training and validation patches, together with 35 test patches, were developed. Using three different breast radiologists, each of the 35 patches in the test set was subdivided in order to assess how well the radiomic characteristics held up through several annotations. An illustration of how the first augmentation strategy generates training image patches. The mass of each individual object in each row is represented along nine different planes. It is divided into nine planes, three of which correspond to the coronal, three of which correspond to the sagittal, and three of which correspond to the axial views, and the remaining six planes correspond to the symmetry planes. The second augmentation technique makes use of the traditional rotation, mirroring, and shearing techniques. Following the affine modifications that were performed in a cumulative method on each mass, 324 patches were created for each of the masses studied.

### 4.2. Performance Evaluation

After the method was trained using all of the supplied data, the average DICE is 0.94 and the conformance was 0.86. However, simply applying the nine planes resulted in much lower classification performance compared to using Affine transformations to increase performance. Improved classification accuracy was achieved by the use of Affine transformations, which outperformed synthetic images (in Figures 2–6).

When comparing the radiomic properties of each radiologist with the classification, the process remained stable. At least 90% of the descriptors remained steady, even when all radiomic features were taken into consideration. However, the percentage of stable features decreased as the correlation criterion was lowered in order to eliminate features that were significantly associated, yet the majority of features remained stable across all comparisons.

Deep learning-based methods were developed for CT imaging. The methods were tested on a large number of expert manual annotations to determine their classification performance. In order to achieve the best classification results, extensive data augmentation was used, including the usage of synthetic images generated by DenseNet. Even while common classification techniques such as rotation and shearing considerably improved classification results. The addition of synthetic examples only increased the DICE findings by 1.3%. DICE rose by 20% when synthetic images were just added, suggesting that DenseNet can still be beneficial in improving classification performance even with small datasets (as demonstrated in this experiment).

Although previous studies on lung classification from chest X-rays found that adding synthetic images to original instances had little impact on classification performance, we believe our results may higher classicization of structures of varying sizes and shapes than or DenseNets. Due to the increasing complexity of classification, it appears that using synthetic images to train a supervised classification model is preferable in circumstances where there are few datasets. Because the conclusions of this study are based on a specific model that was utilized in this investigation, they may be different if alternative designs are used. Therefore, in order to conduct a more relevant performance comparison assessment in the future, new statistics containing additional mass instances will be required, even after accounting for the extremely small boost in classification performance. Because there were only a limited number of mass samples available, the dataset trains the DenseNet algorithms. Synthetic images may have less of an impact on classification performance as a result; classification performance may be enhanced if DenseNet is trained on samples than the model that was used for classification.

It was necessary to rely on a tiny dataset for this investigation, which could have been enhanced by gathering and incorporating additional patient images. As a result of the greater realism in synthetic images, the automatic classification could be improved as a result of the increased realism. It is possible that with larger image datasets, DenseNet architectures based on mask priors, rather than just random noise, will be possible to implement. This would allow for the installation of DenseNet on a conditional basis. Because of the larger input dimensions and pixel level restrictions imposed by the input mask, this technique is more difficult to train, but the quality of the output images may be increased as a result of the larger input dimensions and pixel level restrictions.

By using the DenseNet, we were able to match the training instances, which had an overall total of 450 mass patches, by using the DenseNet. In order to investigate the possibility of an increase in classification performance when the network is taught. Although it is conceivable to incorporate more synthetic cases, we do not anticipate seeing any significant gains because the DenseNet was trained using images from the same set of images that were used to train the U-Net. The usage of more instances to train the DenseNet, particularly examples that are different from those used to train the U-Net, may provide greater insights into the network behavior.

In this work, it was discovered that DenseNet applied to classification in CT scans beat standard unsupervised algorithms, despite the fact that a prior study had been conducted on a different dataset, which may have influenced the results. This method was outperformed by deep learning-based classification algorithms employed in breast ultrasonography, although digital mammography performed comparably to this method. Because breast CT images are in three dimensions, it is possible that U-net training sets will be expanded to include a significantly greater number of examples, possibly due to the higher contrast of the images and the ability to perform significant data augmentation.

There was a significant correlation between the descriptors of distinct categories, indicating that the combination of radiomic descriptors from multiple categories results in a potent signature when used together. Our study indicates that even though the descriptors are recovered from CT lesions have a nonnegligible degree of variability, they have a high degree of robustness, demonstrating that the classification are inconsistent. Furthermore, even after deleting characteristics that were highly associated with the descriptors, the fraction of stable descriptors remained high. When there are a large number of features to examine, overfitting of any predictive model based on feature values is more likely to occur. It is possible to avoid this by simply decreasing the number of features available. However, because our dataset is not sufficiently representative, some features may exhibit low stability despite the good discriminant power of the DenseNet algorithm.

## 5. Conclusions

A detection module is used in conjunction with lengthy training and testing to construct a dense convolutional neural network model. In order to ensure that the model operates as effectively as possible when utilized in cancer detection, various aspects have been incorporated into the design. CT scans are preprocessed in order to obtain the most accurate classification possible during the testing phase. The accuracy of the model in detecting cancer is tested using a 10-fold cross-validation procedure. The experimental validation of the model effectiveness is carried out with the help of Python. When applied to large image datasets, the model outperforms novel approaches in terms of cancer detection. Simulation results indicate that when comparing the suggested method to existing methods, the proposed method has a lower rate of false positives when it comes to detecting cancer. Because the training set is annotated, the classification results may be biased in favor of that radiologist area of expertise. From a radiomics perspective, it appears that this has no significant impact on diagnostic power, but classification performance may be enhanced even further by using the entire dataset, which has been reported on multiple times. In future aspects, we can improvise the methods with the several other deep learning algorithms.

## Figures and Tables

**Figure 1:** Proposed model.

**Figure 2:** Accuracy.

**Figure 3:** Precision.

**Figure 4:** Recall.

**Figure 5:** *F*-measure.

**Figure 6:** MAPE.

## Data Availability

The data used to support the findings of this study are included within the article. Further data or information is available from the corresponding author upon request.
